The article "The Conditioned Medium of Lactobacillus rhamnoides GG Regulates Microglia/Macrophage Polarization and Improves Functional Recovery after Spinal Cord Injury in Rats" was retracted in 2024. Reasons: signs of a paper mill; suspected computer-generated content; unreliable results or conclusions; concerns about the data.

# The Conditioned Medium of Lactobacillus rhamnoides GG Regulates Microglia/Macrophage Polarization and Improves Functional Recovery after Spinal Cord Injury in Rats

**DOI:** 10.1155/2021/3376496

**Published:** 2021-07-10

**Authors:** Fangqi Lin, Baokun Zhang, Qiang Shi, Jiaming Liang, Xin Wang, Xiaofeng Lian, Jianguang Xu

**Affiliations:** Department of Orthopedic Surgery, Shanghai Jiao Tong University Affiliated No.6 People's Hospital, 600 Yishan Road, Shanghai 200233, China

## Abstract

Lactobacillus rhamnoides, a human intestinal colonizer, can act through various pathways to induce microglia/macrophages to produce cytokines and to polarize microglia/macrophages to different phenotypes to reduce the inflammatory response. In this article, we evaluated the treatment potential of the Lactobacillus rhamnoides GG conditioned medium (LGG-CM) in rat model with SCI (acute spinal cord injury), including functional, neurophysiological, and histological outcomes and the underlying neuroprotective mechanisms. In our experiment, LGG-CM (30 mg/kg) was injected directly into the injury site in rats immediately after SCI. Measured by the BBB scale (Basso, Beattie, and Bresnahan locomotor rating scale) and inclined plane test, rats in the LGG-CM-treated group showed better locomotor scores. Moreover, compared to the vehicle treatment group, LGG-CM increased the mRNA level of the M2 marker (CD206), and decreased that of the M1 marker (iNOS). Western blot assays showed that LGG-CM-treated SCI rats had a higher grayscale ratio of p65 and a lower ratio of p-I*κ*B*α*/I*κ*B*α*. Our study shows that local injection of LGG-CM after acute SCI can inhibit inflammatory responses and improve motor function recovery. These effects may be related with the inhibition to the NF-*κ*B (The nuclear factor-kappa B) signal pathway which leads to M2 microglia/macrophage polarization.

## 1. Introduction

SCI (spinal cord injury), which is often secondary to spinal injury, is the most severe complication of spinal trauma and often leads to serious limb dysfunction [1]. SCI can cause local tissue destruction and microcirculation disturbances, resulting in the exacerbation of local damage and extensive necrosis of peripheral nerve cells, which in turn can cause motor, sensory, and autonomic dysfunction in the human body, greatly reducing the quality of life of patients [2, 3]. A previous study has proved that timely medication and intervention after spinal cord injury can attenuate long-term functional impairment and pathological damage [4]. So it is essential to develop effective methods to promote locomotor function recovery after SCI. Methylprednisolone is currently most commonly used clinically, but it must be carefully monitored to prevent arrhythmia, circulatory failure, and cardiac arrest, as well as complications of gastrointestinal bleeding [5]. Other drugs such as naloxone, nerve growth factor, and thyrotropin-releasing hormone have been shown to be effective in the recovery of spinal cord function in experiments, but they have yet to be confirmed by their extensive clinical application [6–8].

Within a few hours after spinal cord injury, microglia/macrophages, as the first immune cells to react to injury, polarize into M1 microglia/macrophages, releasing inflammatory factors (TNF-*α*, IL-6, and IL-1*β*), exacerbating the inflammatory response, inhibiting axonal regeneration, and finally leading to apoptosis of residual neurons [9, 10]. At later stages of spinal cord injury, the inflammatory response gradually weakens, and inflammatory factors secreted by M1 microglia/macrophages gradually decrease, and M2 microglia/macrophages play a key gradually. M2 microglia/macrophages can make regeneration and functional recovery of residual nerves by modifying the microglia/macrophage phenotype, reducing the secretion of proinflammatory factors, increasing the secretion of neurotrophic factors, and increasing stimulatory factors in the microenvironment, such as TGF-*β*1 [11, 12]. The predominance of the M1 phenotype instead of M2 phenotype after SCI may contribute to secondary damage of the spinal cord. But, it is still unclear which factors in SCI can lead to microglia/macrophage phenotype switching. The switch of microglia/macrophage has been successfully applied in the treatment of chronic inflammatory renal disease, type 1 diabetes, and autoimmune encephalomyelitis in animal models [13–17], but the reports about this method applied in SCI treating are yet not so complete.

Lactobacillus rhamnoides, a kind of Gram-positive bacterium, can produce a large amount of lactic acid from fermentable carbohydrates [18]. Moderate intervention to the NF-*κ*B signal pathway can reduce inflammatory response. Studies have shown that the conditioned medium of Lactobacillus rhamnoides GG (LGG-CM) can promote microglia/macrophage polarization to M2 by inhibiting the NF-*κ*B signal pathway; this has been proven in the context of Salmonella infantis-induced inflammation in a pig model and colitis in mice [19, 20]. However, it has not been reported whether lactic acid bacteria can promote the repair of SCI by regulating the polarization of microglia/macrophages. Given its ability to regulate cytokines secreted by microglia/macrophages and microglia/macrophage polarization, we used LGG-CM in the treatment of SCI rats for the first time, to investigate whether it can reduce the nerve damage caused by SCI and promote the recovery of behavioral motor function.

## 2. Materials and Methods

### 2.1. Ethical Approval

All rats were operated on by the same surgeon. The animals were anesthetized by using 30 mg/kg pentobarbital administered intraperitoneally. The anesthetic effect was expected to begin within 5 min and to last approximately 2 hours, which was enough time to complete the spinal cord injury procedure. The withdrawal reflex to tail compression was used to evaluate the level of anesthesia.

### 2.2. Drugs

Lactobacillus rhamnoides was inoculated in MRS medium and cultured for 24 h at 37°C. We centrifuged the supernatant and filtered out the bacteria with a 0.22 *μ*m filter membrane, loaded them into an enrichment tube, and centrifuged them at 4000 r/min for 40 min at 4°C. From previous studies, we can know that the active ingredient of LGG-CM has a relative molecular weight ≥ 30000 kDa, and our preexperimental results also showed that the LGG-CM component with a relative molecular weight ≥ 30000 kDa significantly promoted microglia/macrophage polarization from M1 to M2 state. Therefore, we used the LGG-CM component with a molecular weight of ≥30000 kDa in this study.

### 2.3. Animals

Female rats (200–220 g, approximately 2 months) were reared in cages (every cage had 4 rats) in an environment with controlled temperature (25°C) and light/dark cycle (12/12 h). All rats had sufficient water and food during the whole study, and we made lots of efforts to alleviate the rats' suffering.

The rats were divided into the 3 groups randomly, in which SCI or laminectomy was performed. In clinical practice, some doctors inject methylprednisolone into the local area of nerve decompression surgery and administer it in the form of local infiltration, which has played a good auxiliary role in surgical treatment. Similarly, the mice were directly administered LGG-CM (30 mg/kg) or saline at the site of injury by intrathecal injection within the first hour. The animal groups were as follows:

1. SCI+saline (SCI+vehicle)
2. SCI+2 ml/kg LGG-CM (SCI+LGG-CM)
3. Sham+saline (sham; same surgical operation as the other 2 groups, except that weight dropping to the dura was not applied)

At 1, 2, 3, 4, 5, 6, and 7 days postsurgery, each rat was subjected to behavioral function assessment. And at 1, 3, and 7 days after surgery, we sacrificed 3 rats from each group and excised their spinal cords for follow-up biochemical studies and staining.

### 2.4. In Vitro Experiments

#### 2.4.1. Cell Counting Kit-8

The degrees of cell viability of different LGG-CM concentrations were assessed with CCK-8 (Cell Counting Kit-8). Briefly, LGG-CM (LGG-CM: PBS (phosphate buffer saline) at 4 concentrations: 0, 1 : 100, 1 : 50, and 1 : 25) was added to 96-well plates, and each well was seeded with 200 *μ*l cells at a concentration of 1 × 10^4^ cells/ml. Incubated for 0 and 24 hours, the cells were added with 10 *μ*l CCK-8 reagent. Then, the plates would be incubated for 1 hour. Finally, we used a microplate reader to measure spectrophotometric absorbance at 450 nm.

#### 2.4.2. Flow Cytometric Measurement

THP-1 cells were incubated or differentiated in media containing different concentrations of LGG-CM (0 *μ*l/ml, 10 *μ*l/ml, and 20 *μ*l/ml). The microglia/macrophages were detached with trypsin. The collected microglia/macrophages were washed twice in PBS (phosphate buffer saline) and then resuspended in PBS again at a concentration of 1 × 10^7^ cells/ml. We transferred 100 *μ*l of suspended cells to a flow tube. After that, we stained the cells with fluorescent dye-conjugated antibodies against CD206, CD86, and the corresponding isotype controls at 4°C. Washed twice in PBS again, the stained cells were then analyzed by FACSAria flow cytometry on a flow cytometer. The software we used for analyzing results was FlowJo. Flow cytometry and fluorescence microscopy were used to measure apoptosis. We used PBS to wash the cells twice and then used trypsin to detach. We centrifuged the THP-1 cells at 1000 rpm for 3 min, washed them in PBS twice, and added Annexin V Binding Solution (1×) to the cells, which were maintained at a fixed concentration of 1 × 10^6^ cells/ml; then, we transferred 100 *μ*l of the cell-containing solution to prepared flow tubes. We added FITC Annexin V (5 *μ*l) and propidium iodide (PI, 5 *μ*l) to each tube, incubated the tubes for 15 min in the dark, and then added 400 *μ*l of 1× Annexin V Binding Solution to each tube. The results were analyzed by a FACSAria flow cytometer and fluorescence microscopy.

### 2.5. In Vivo Experiments

#### 2.5.1. Animal Surgery

Animals were anaesthetized by pentobarbital (30 mg/kg body weight). After the hair at the surgical area was shaved, the skin of the surgical area was disinfected with medical alcohol (70%) and povidone-iodine. Under aseptic conditions, we made a longitudinal incision on the midline of the rat back to expose the paravertebral muscles. The T5–T8 vertebrae were exposed after dissecting the paravertebral muscles away. After exposing the spinal cord by T5-T8 laminectomy, we performed extradural compression by dropping a rod (diameter: 2 mm; weight: 10 g; height: 20 mm) to the dura rapidly to produce SCI. The rats in the sham group were only subjected to laminectomy. Ten minutes after SCI, rats in the LGG-CM group were administered direct injections of LGG-CM (2 ml/kg) at the injured segment of the spinal column, and the same volume of PBS was injected into rats in the vehicle group. We set the pH of the LGG-CM solution at between 7.2 and 7.4 to match the normal tissue pH. To replenish the blood lost in the surgery, 1 ml of saline was injected subcutaneously. The rats were placed in an area with warm heating lights during the recovery from anesthesia. During the whole experiment, sufficient food and water were provided. We manually voided rat bladders twice daily until bladder function returned to normal.

#### 2.5.2. Basso, Beattie, and Bresnahan Locomotor Rating Scale

We used the BBB scale (Basso, Beattie, and Bresnahan locomotor rating scale) to evaluate the locomotor function of rats. Based on paw placement, limb movement, coordination and gait, the BBB scale is a detailed classification system of functional scores ranging from 0 to 21 (0 for no hindlimb movement and 21 for normal hindlimb movement) [21]. From day 1 to day 7 after the surgery, each rat was observed by at least two different experimenters who were blinded to the treating methods received for each rat. During a 5 min walk, the rats were positioned in an open and smooth field so that they could be observed on both sides.

#### 2.5.3. Inclined Plane Test

We used an inclined plane test to assess the muscle strength of the rat hind paws [22]. The rats were observed and evaluated by two different experimenters who were blinded to the treating methods received for each rat. The rats were placed on an inclined plane that was then gradually raised from 0° by 1° at a time, and the maximum angle at which the rat could remain on the inclined plane was observed. Each rat was tested at least 3 times, and the data would be averaged for subsequent analysis.

#### 2.5.4. Tissue Preparation

At 1, 3, and7 days post-SCI, the rats were sacrificed with overdose pentobarbital (100 mg/kg; Nembutal). The rats, whose spinal cords would be used for staining, were perfused transcardially with cold normal saline and 4% paraformaldehyde in sequence. After careful dissection, the spinal cords were fixed in 4% paraformaldehyde at 4°C overnight, dehydrated with 30% sucrose, embedded in paraffin wax, and then sectioned (5 *μ*m). For the spinal cords which were used for PCR and Western blot analysis, we made a dissection for segments of approximately 1 cm concluding the area of injury, washed them with PBS (ice-cold phosphate-buffered saline), and then snap-frozen and stored in liquid nitrogen until analysis.

### 2.6. Hematoxylin-Eosin Staining and Nissl Staining

We stained the spinal cord sections (20 *μ*m) with conventional hematoxylin-eosin (H&E) staining and Nissl staining and observed the stained sections through an optical microscope. In hematoxylin-eosin staining, after deparaffinization and rehydration, we stained 5 *μ*m longitudinal sections with hematoxylin solution for 5 min, then immersed the sections in 1% acid ethanol (1% HCl in 70% ethanol) solution, and then rinse in distilled water totally. Then, the sections were stained with eosin solution for 3 min, and then dehydrated with gradient alcohol and clarified in xylene. In Nissl staining, we first heated the sections at room temperature for 30 min, then immersed the sections in 100% ethanol, 75% ethanol and distilled water for 30 seconds, and then stained them with 0.1% cresyl violet solution at 37°C for 5 min. After the sections were completely washed in distilled water, they would be immersed in 95% ethanol for 30 seconds and then immersed in absolute ethanol, absolute ethanol, and xylene for 5 minutes. Finally, seal the sections with neutral glue and observe under a microscope.

### 2.7. Immunohistochemistry

Spinal cord sections were stained for: MMPs (matrix metalloproteinases). After fixation, the sections were washed with PBST (30 min) and then incubated in normal goat serum (10%, 30 min) for blocking. The transverse sections were then incubated with the primary antibodies MMPs, at 4°C for 12 h. Subsequently, the sections were washed again in PBST (30 min) and then incubated with the secondary antibodies for 8 h. Finally, the sections were washed with PBST (30 min) and then incubated with DAPI for 30 s and cover-slipped. Images were captured by a laser scanning confocal microscope. Three consecutive slices from each animal were analyzed, and three random visual fields were counted in each slice.  Table 1 shows the information of antibodies.

### 2.8. Real-Time PCR

Following the standard manufacturer's instructions, we used an RNA simple total RNA kit to isolate total RNAs from the injured spinal cords. The concentration and quality of total RNA were assessed by spectrophotometric determination at 260/280 nm, and equal amounts of RNA from each sample were reverse-transcribed into complementary DNA (cDNA) for RT-qPCR. For miRNA reverse transcription, cDNA was synthesized using the miRNA First-Strand cDNA Synthesis (Tailing Reaction) Kit (Sangon Biotech, Shanghai). For mRNA reverse transcription, cDNA was synthesized using the PrimeScript RT Reagent Kit with gDNA Eraser (TaKaRa Biomedical Technology Co. Ltd., Beijing, China). cDNA was further applied as a template for RT-qPCR following the manufacturer's instructions (Mastercycler Gradient; Eppendorf, Germany). The primers are shown in Table 1.

### 2.9. Western Blot Analysis

Microglia/macrophages isolated from mice treated with or without LGG-CM were homogenized with ice-cold RIPA buffer (25 mM Tris-HCl pH 7.6, 150 mM NaCl, 1% NP-40, 1% sodium deoxycholate, and 0.1% SDS) containing protease and phosphatase inhibitors (Complete Protease Inhibitor Cocktail and PhosSTOP Phosphatase Inhibitor Cocktail; both from Roche). After centrifugation at 12,000 g for 10 min at 4°C, the supernatants were collected. The protein concentration was determined using a bicinchoninic acid (BCA) assay (QuantiPro BCA Assay Kit, Sigma-Aldrich) according to the manufacturer's instructions. Protein samples were separated by SDS-polyacrylamide gel electrophoresis and transferred onto polyvinylidene fluoride (PVDF) membranes (Millipore Corporation, USA). The membranes were blocked with 5% skimmed milk for 1 h at room temperature and then incubated with primary antibodies at 4°C overnight: rabbit anti-p-I*κ*B*α* (1 : 1000; Cell Signaling Technology), rabbit anti-I*κ*B*α* (1 : 1000; Abcam), and rabbit anti-*β*-actin (1 : 1000; Abcam). After three washes, the members were incubated with an HRP-coupled secondary antibody (1 : 20000; Jackson) at room temperature for 1 h and washed three times for 10 min each at room temperature. Finally, all the membranes were imaged using densitometry (ChemiScope 6100) and quantified using densitometric analysis (ImageJ software, NIH).

### 2.10. Statistical Analysis

We used GraphPad Prism software 8.0 to perform statistical analysis. Two-tailed unpaired Student's *t*-test was used to compare the two groups. Unless otherwise stated, the rest of the data were analyzed by either one-way or two-way analysis of variance with post hoc Tukey's multiple comparisons tests. *P* values of < 0.05 were considered significant.

## 3. Results

### 3.1. Experimental Protocol

The scheme of our article explains the protocol (Figure 1).

### 3.2. Cell Survival Assay

To determine the appropriate dose of LGG-CM, microglia/macrophage cells were incubated with 0 (control), 1 : 25, 1 : 50, and 1 : 100 LGG-CM : PBS for 24 h. We can find from the CCK-8 results assay that LGG-CM significantly increased cell viability compared to the control. The 1 : 50 concentration had a greater effect on viability than the other concentrations and also promoted the most microglia/macrophage polarization to M2. Thus, 1 : 50 (20 *μ*l/ml) was selected for use in the subsequent experiments (Figure 2).

### 3.3. LGG-CM Improves Functional Restoration after Acute SCI

We performed BBB and inclined plane tests daily from 1 to 7 days after SCI to evaluate the functional restoration of mice in different groups. As the higher BBB scores indicated, the LGG-CM-treated group showed improved recovery from day 3 after SCI. Compared to the rats of the vehicle-treated group, the rats of the LGG-CM-treated group showed better locomotor function recovery in inclined plane test, with a significantly increased angle of the inclined plane that the rats could stay (Figure 3).

### 3.4. LGG-CM Reduces Lesion Size

At 7 days post-SCI, the area of spinal cord damage on the specimens in the LGG-CM-treated group was noticeably less than that in the vehicle-treated group. Moreover, Nissl staining suggested that the density of Nissl bodies in the LGG-CM-treated group was significantly higher than that in the vehicle-treated group at 7 days after SCI (Figure 4).

### 3.5. LGG-CM Polarization to M2 Microglia/Macrophages and Reduce Inflammation

At 7 days after surgery, we used immunochemistry and immunofluorescence staining to observe the spinal cord slices of rats with spinal cord injury to study the changes of matrix metalloproteinases (MMPs) near the slices. We found that the expression of MMPs was low in the sham group. In both the LGG-CM group and vehicle group, the expression of MMPs was higher than that in the sham group significantly; the expression of MMPs was less in the LGG-CM compared with the vehicle group. Then, we used qPCR to value the mRNA levels of MMP-9 and characteristic surface markers (TNF-*α*, IL-6, IL-1*β*, TGF-*β*1, CD206, and iNOS) at day 7 after surgery. As expected, LGG-CM treatment reduced the mRNA expression of MMP-9, iNOS, IL-6, IL-1*β*, and TNF-*α*. On the contrary, the mRNA expression CD206 and TGF-*β* was significantly increased in LGG-CM-treated rats. The mRNA marker expressions of both M1 and M2 in the vehicle-treated group were significantly higher than that in the sham group. Compared to vehicle treatment, LGG-CM treatment can increase the mRNA expression of M2 markers and decreased that of M1 markers (Figure 5).

### 3.6. LGG-CM Inhibits the NF-*κ*B Signal Pathway by Reducing the Phosphorylation of I*κ*B*α*

The NF-*κ*B (nuclear factor-kappa B) signal pathway is crucial in the process of producing inflammatory cytokines to perform proinflammatory functions. We hypothesized that LGG-CM can protect rats against SCI by inhibiting NF-*κ*B-mediated inflammation. To verify our hypothesis, we used immunoblotting to assess the NF-*κ*B activation and assessed the expression of NF-*κ*B in microglia/macrophages by immunostaining. In the LGG-CM treatment group, we could observe an inhibition of NF-*κ*B p65, suggesting that LGG-CM can suppress the transcriptional activity of NF-*κ*B p65. Moreover, the ratio of p-I*κ*B*α*/I*κ*B*α* was significantly lower in rats with LGG-CM treatment, which means that the NF-*κ*B signaling pathway was inhibited by reducing the phosphorylation of I*κ*B*α* (Figure 6).

## 4. Discussion

After ensuring the safety of LGG-CM by CCK-8 test and the effectiveness by flow cytometric measurement, we applied LGG-CM locally at the injured site after SCI in rats. From the observation of the treatment group, we can find a less damage area of spinal cord specimens and a higher density of Nissl bodies. Evaluated by BBB test and inclined plane test, functional recovery was improved significantly in the treatment group, which shows that LGG-CM do provide a protective effect against SCI in rats. The results of PCR and Western blot experiments showed that the therapeutic effect was associated with the inhibition of the NF-*κ*B signal pathway, which promoted the polarization of microglia/macrophages to M2 rather than M1 and thereby reduced related inflammatory processes and improved locomotor function recovery.

With the mediation of inflammatory mediators, matrix metalloproteinases (MMPs) can cause the dissolution of extracellular matrix and the destruction of basement membrane, aggravating the inflammatory response and destroying normal cell tissues. What is more, the expression of MMPs is positive with the inflammatory mediators. So MMPs can be used to assess the severity of inflammatory response [23–25]. From the results of immunohistochemistry and immunofluorescence staining, we found that in the sham operation group, the expression of MMPs was low, which is in line with the description in the literature review: the expression of MMPs in normal tissues was low or even not expressed. In the LGG-CM group and the vehicle group, the expression of MMPs was higher than that in sham group, and the expression of MMPs in the LGG-CM group was lower than that in the vehicle group. This indicates that the intervention of LGG-CM can reduce the inflammatory response of spinal cord injury tissue, and its effect may be related to the reduction of inflammatory mediators.

The inflammatory response plays an important role during the process of local tissue injury after SCI. In well-defined in vitro situations, microglia/macrophages can be divided into the M1 (proinflammatory) phenotype and M2 (anti-inflammatory) phenotype by the presence of different surface markers. The dominance of the M1 or M2 phenotype can determine the trend of immune responses [26]. The proinflammatory M1 state may be related to the dominant expression of proinflammatory factors (TNF-*α*, IL-6, IL-1*β*, and iNOS) that exacerbate local inflammation. On the contrary, the anti-inflammatory M2 state is associated with the dominance of anti-inflammatory factors (TGF-*β*1 and CD206), which is beneficial for tissue repair [27, 28]. In our research, we observed the changes of inflammatory factors and microglia/macrophage markers by real-time PCR. We can find that in the first few hours after SCI, microglia/macrophages polarized to the M1 phenotype, and proinflammatory factors increased and remained a high level for 3 days after SCI. In the late stage of SCI, microglia/macrophages polarized to M2, with a significant increase of anti-inflammatory factors (i.e., TGF-*β*1 and CD206). These results offer a possible therapeutic strategy that regulates the polarization of microglia/macrophages to decrease excess neuroinflammatory factor levels and block inflammatory responses which may downregulate the production of inflammatory cytokines and inhibited inflammation, to promote neural functional repair after SCI.

LGG is currently one of the most widely studied probiotics, and it has been proven effective in preventing and treating certain conditions, such as intestinal infections, diarrhea, systemic inflammation, and allergic diseases [29, 30]. Studies have shown that LGG-CM can reduce intestinal damage caused by pathogenic bacteria and oxidative stress [31, 32]; moreover, LGG-CM reduced allergic reactions and enhanced the immune function of mononuclear microglia/macrophages when administered to mice [33, 34]. In a previous study, it was found that LGG-CM can directly act on brain microvascular cells to inhibit the activation of the NF-*κ*B signal pathway. [35] We applied LGG-CM to SCI rats and found that LGG-CM can reduce the occurrence of inflammation in SCI and do exert a therapeutic effect. During in vitro experiments, we ensured the safety of LGG-CM by CCK-8 test. And then, we treated microglia/macrophages with different concentrations of LGG-CM and found that the effect of LGG-CM on polarization was concentration dependent. From the real-time PCR results, we can find that compared to vehicle treatment, LGG-CM treatment significantly decreased the mRNA levels of M1 state markers (iNOS) near the injury section of SCI rats, which shows that LGG-CM administration may inhibit polarization to M1. Conversely, the mRNA levels of markers of M2 were increased, which means that polarization to M2 was promoted. As indicated by our behavioral analyses, LGG-CM can promote the polarization of microglia/macrophage to M2 phenotype rather than M1 phenotype and thus improve the recovery of motor function.

In fact, the dominance of the M1 or M2 phenotype in vivo may be associated with many conflicting factors from the physiological environment. As a key transcription factor, NF-*κ*B plays an important role in microglia/macrophage polarization. NF-*κ*B pathways are activated by extracellular stimuli. Extracellular signaling factors bind to the corresponding receptors on the cell membrane, initiating a series of downstream responses. The stimulated receptor protein activates I*κ*B kinase (IKK). IKK phosphorylates the serine within the amino-terminal domain of I*κ*B in the intracellular NF-*κ*B I*κ*B complex so that the I*κ*B subunit is modified by ubiquitination and then degraded by proteases, thereby releasing the NF-*κ*B dimer. The activated NF-*κ*B dimer is mainly composed of the p50 subunit and p65 subunit. In the NF-*κ*B pathway, the activation of p65 can initiate inflammation in the human body and induce microglia/macrophage polarization to M1. Our Western blot assay indicated that the grayscale ratio of p65 was lower in the LGG-CM-treated SCI rats, suggesting that LGG-CM can inhibit the transcriptional activity of NF-*κ*B p65. Moreover, the ratio of p-I*κ*B*α*/I*κ*B*α* was significantly lower in LGG-CM-treated SCI rats, which indicates that the phosphorylation of I*κ*B*α* was reduced. Collectively, these findings suggest that LGG-CM inhibited the NF-*κ*B pathway by reducing the phosphorylation of I*κ*B*α*, which can promote microglia/macrophage polarizing to the anti-inflammatory M2 state to repair injury tissue and reduce inflammation.

## 5. Conclusion

Our study suggests a novel treatment strategy: early LGG-CM administration immediately after SCI reduced the extent of posttraumatic inflammation near the injured site and promoted locomotor function recovery after SCI. This occurred through a mechanism in which LGG-CM inhibited the NF-*κ*B pathway by reducing the phosphorylation of I*κ*B*α*, which promoted microglia/macrophage polarization to M2 and inhibited polarization to M1. Thus, LGG-CM is expected to be a candidate therapeutic drug for exerting neuroprotection after SCI.

## Figures and Tables

**Figure 1:** The scheme of our article.

**Figure 2:** (a, b) Cell viability of in different percentage of LGG-CM and PBS at 0 h and 24 h (NC, 1 : 100, 1 : 50, and 1 : 25). (c–e) Flow cytometric measurement. (f) The expression of Arg-1 and CD206 at different concentrations of LGG-CM (NC, 10 *μ*l/ml, and 20 *μ*l/ml).

**Figure 3:** LGG-CM treatment promotes the recovery of locomotor functions after SCI. (a–d) Quantification of BBB score from day 1 to day 7 after surgery. (e–h) Quantification tested by inclined plane test from day 1 to day 7 after surgery.

**Figure 4:** LGG-CM attenuates tissue damage. (a) H&E staining of transverse spinal cord sections near the injury at day 7 after SCI. (b) Nissl staining of transverse spinal cord sections near the injury at day 7 after SCI. (c) The area of injury site in SCI rats who were treated with LGG-CM or vehicle. (d) Quantification of lesion as a ratio to whole area at the epicenter in each SCI group. (e) Numbers of Nissl bodies (/mm^2^) in transverse spinal cord sections near the injury at day 7 after SCI.

**Figure 5:** LGG-CM treatment reduces neuroinflammation in the spinal cord after SCI. (a) Immunohistochemistry and immunofluorescence images of MMPs in the spinal cord at 7 days post-SCI. (b–e) The mRNA levels of iNOS (b), IL-6 (c), IL-1*β* (d), and TNF-*α* (e) near the injury section at day 7 post-SCI of the sham operation, SCI+vehicle, and SCI+LGG-CM treatments. (f, g) The mRNA levels of TGF-*β*1 (f) and CD206 (g) near the injury section at day 7 post-SCI of the sham operation, SCI+vehicle, and SCI+LGG-CM treatments. (h) Upregulation of MMP-9 activity after SCI is demonstrated. After LGG-CM treatment, the activity was downregulated.

**Figure 6:** LGG-CM treatment could inhibit NF-*κ*B signal pathway by reducing the phosphorylation of I*κ*B*α*. (a) Western blot images show the expression of I*κ*B*α*, p-I*κ*B*α*, and p65 in microglia/macrophage. (b, d, f) The grayscale ratio of I*κ*B*α* in the spinal cord of mice at 1 (b), 3 (d), and 7 (f) days post-SCI. (c, e, g) The grayscale ratio of p65 in the spinal cord of mice at 1 (c), 3 (e), and 7 (g) days post-SCI. (i–k) The grayscale ratio of p-I*κ*B*α* in the spinal cord of mice at 1 (i), 3 (j), and 7 (k) days post-SCI. (h) The ratio of p-I*κ*B*α*/I*κ*B*α* in the spinal cord of mice.

**Table 1:** Primers used for real-time PCR.

Genes	Forward primers	Reverse primers
*β*-Actin	5′ CCT CTA TGC CAA CAC AGT 3′	5′ AGC CAC CAA TCC ACA CAG 3′
IL-6	5′ AAT CTG CTC TGG TCT TCT GGA 3′	5′ ATT GCT CTG AAT GAC TCT GGC 3′
IL-1*β*	5′ GTT CTT TGA GGC TGA CAG ACC 3′	5′ GAT GCT GCT GTG AGA TTT GAA 3′
TNF-*α*	5′ CCA ATC TGT GTC CTT CTA ACT 3′	5′ TGT GTT TCT GAG CAT CGT 3′
iNOS	5′ CTC AGG CTT GGG TCT TGT TAG 3′	5′ TCT GTG ACT TTG TGC TTC TGC 3′
CD206	5′ CCT TCT GTG CCT ATC TCT CCA 3′	5′ TAT TTC TCT GCT TCG TGC CAT 3′
TGF-*β*1	5′ CCT GGA TAC CAA CTA CTG CTT 3′	5′ AGG TCC TTC CTA AAG TCA ATG T 3′
MMP-9	5′ GAC TCG GTC TTT GAG GAG CC 3′	5′ GAA CTC ACG CGC CAG TAG AA 3′

## Data Availability

The data used to support the findings of this study are included within the article.
